# Alpha-Fetoprotein Promoter-Driven Cre/LoxP-Switched RNA Interference for Hepatocellular Carcinoma Tissue-Specific Target Therapy

**DOI:** 10.1371/journal.pone.0053072

**Published:** 2013-02-28

**Authors:** Yuan-Fei Peng, Ying-Hong Shi, Zhen-Bin Ding, Jian Zhou, Shuang-Jian Qiu, Bo Hui, Cheng-Yu Gu, Hua Yang, Wei-Ren Liu, Jia Fan

**Affiliations:** 1 Department of Liver Surgery, Liver Cancer Institute, Zhongshan Hospital, Fudan University; Key Laboratory of Carcinogenesis and Cancer Invasion of Ministry of Education, Shanghai, People's Republic of China; 2 Institutes of Biomedical Sciences, Fudan University, Shanghai, People's Republic of China; University of Alabama at Birmingham, United States of America

## Abstract

**Backgroud:**

RNA interference (RNAi) has recently emerged as a potential treatment modality for hepatocellular carcinoma (HCC) therapy, but the lack of cellular targets and sustained efficacy limits its application. The purpose of this study is to develop an HCC tissue-specific RNAi system and investigate its possibility for HCC treatment.

**Methods:**

Two different HCC-specific RNAi systems in which therapeutic miRNA or shRNA against target gene (Beclin 1) was directly or indirectly driven by alpha-fetoprotein promoter (AFP-miRNA and AFP-Cre/LoxP-shRNA) were constructed. Human HCC cell lines (HepG2, Hep3B and HCCLM3) and non-HCC cell lines (L-02, Hela and SW1116) were infected with the systems. The effectiveness and tissue-specificity of the systems were examined by Q-PCR and western blot analysis. The efficacy of the systems was further tested in mouse model of HCC by intravenous or intratumoral administration. The feasibility of the system for HCC treatment was evaluated by applying the system as adjuvant therapy to enhance sorafenib treatment. An AFP-Cre/LoxP-shRNA system targeting Atg5 gene (AFP-Cre/LoxP-shRNA-Atg5) was constructed and its efficacy in sensitizing HCC cells (MHCC97L/PLC) to sorafenib treatment was examined by apoptosis assay *in vitro* and tumorigenesis assay *in vivo*.

**Results:**

The AFP-miRNA system could silence target gene (Beclin 1) but required a high titer which was lethal to target cells. The AFP-Cre/LoxP-shRNA system could efficiently knockdown target gene while maintain high HCC specificity. Intratumoral injection of the AFP-Cre/LoxP-shRNA system could efficiently silence target gene (Beclin 1) *in vivo* while intravenous administration could not. The AFP-Cre/LoxP-shRNA system target Atg5 gene could significantly sensitize MHCC97L/PLC cells to sorafenib-induced apoptosis *in vitro* and tumor growth suppression *in vivo*.

**Conclusions:**

An efficient HCC tissue-specific RNAi system (AFP-Cre/LoxP-shRNA) was successfully established. The system provides a usable tool for HCC-specific RNAi therapy, which may serve as a new treatment modality for HCC.

## Introduction

Hepatocellular carcinoma (HCC) is the sixth most common cancer and the third most frequent cause of cancer-related death [1]. The prognosis of HCC is poor for most of patients because HCC is often diagnosed at a late stage and current treatment options are rather limited. The inherent difficulty of treating this malignancy has prompted many to consider new therapeutic approach.

In recent years RNA interference (RNAi) has emerged as a potential treatment modality for cancer therapy. RNAi is a sequence-specific posttranscriptional gene silencing process. Since its discovery, RNAi has been rapidly developed into a powerful technique for both therapeutic and gene functional research. Several clinical trials published so far and numberous *in vivo* animal studies have demonstrated the success and feasibility of RNAi for the treatment of various diseases [2]–[5]. HCC is a disease of altered genes. In recent years, unprecedented advances in genome-wide analysis have resulted in important discoveries regarding HCC. The cancer-causing genes identified by the new genome-wide technologies have provided great opportunities for HCC therapy [6]. In addition, since RNAi can be easily delivered into the liver, HCC is amenable to RNAi targeting and it has been extensively used as a disease model for testing RNAi therapy [5], [7]. Therefore, RNAi therapy has tremendous potential as a treatment modality for HCC therapy. It is foreseeable that RNAi technique will be widely appliedapplicable for HCC treatment in the near future.

However, although RNAi is highly attractive as a therapeutic approach, several hurdles must be overcome before RNAi can be successfully introduced into the clinic. These include efficiency of cellular uptake, specific guidance to target tissue or cell, and sustained efficacy [3]–[5], [8]. The RNAi should be limited to target cells and nonspecific cytotoxicity should be avoided. It is especially important to the RNAi therapy for HCC because HCC frequently occurs in patients with liver cirrhosis and compromised hepatic function reserve. The currently most popular materials used for RNAi are chemically synthesized small interfering RNA (siRNA) and vector-based short hairpin RNA (shRNA) driven by Pol III promoters (U6 or H1). However, either siRNA or Pol III promoter-driven shRNA can silence target gene in all cell types, and therefore may destroy not only target tumor cells but also non-tumor cells. Besides, the duration of siRNA or vector-based shRNA induced silencing was short-term and lasted less than a few weeks [5]. But RNAi therapy usually requires much longer duration of action (in some cases, years). In addition, the *in vivo* cellular uptake and intracellular delivery still remain a major challenge for therapeutic application of RNAi [9]. To obtain tissue-specific, long-term and high efficient RNAi, one possible solution is to employ tissue-specific promoter (to restrict therapeutic RNAi expression in target tissue) in combination with lentiviral vector (to obtain high transduction efficiency and stable gene silencing). One of the major characteristics of hepatocellular carcinoma is the transcriptional reactivation of alpha-fetoprotein (AFP) [10]. The AFP promoter is highly specific to HCC. It has been employed to drive therapeutic gene expression to develop HCC-specific gene therapy, although there have been few reports on its application in RNAi therapy [11]–[16]. The long-term high-efficiency gene silencing required for RNAi therapy can be achieved by using lentiviral vectors. Lentivirus-mediated RNAi is a powerful method for long-term inhibition of gene expression *in vitro* and *in vivo* [17]. The small interfering RNA can be delivered through lentiviral vector in a form of shRNA driven by a Pol III promoter or a miRNA-like structure expressed from a Pol II promoter [17]. The shRNA or miRNA contained in lentiviral vectors can be stably integrated into the genome, which allows permanent, heritable gene silencing. The lentivector technology has been widely used in basic and translational research, and it has been applied in clinic and provides therapeutic benefit [17].

The purpose of this study was to develop an efficient HCC tissue-specific RNAi system and investigate the possibility of the system for HCC treatment. We constructed two different HCC tissue-specific RNAi systems in which therapeutic miRNA or shRNA against target gene (Beclin 1) was directly or indirectly driven by an AFP promoter (AFP-miRNA system and AFP-Cre/LoxP-shRNA system). The effectiveness and tissue-specificity of the systems were examined in HCC and non-HCC cells *in vitro* and *in vivo*. The feasibility of the system as new agent against HCC was tested based on the finding in previous research that silencing Atg5 gene could enhance sorafenib lethality [18]. The HCC tissue-specific RNAi system targeting Atg5 gene was constructed and the efficacy of the system for sensitizing HCC cells to sorafenib treatment was examined *in vitro* and *in vivo*.

## Materials and Methods

### Cell Lines and Animals

Human HCC cell lines Hep3B, HepG2, PLC/PRF/5 (ATCC), HCCLM3 [19], [20], and MHCC97L [20], [21], human normal hepatic cell line L-02 (Cell Bank, China), human cervical carcinoma cell line HeLa and colon cancer cell line SW1116 (ATCC) were routinely maintained. Male BALB/c nu/nu mice (6 weeks old, Chinese Academy of Science) were bred in specific pathogen-free conditions. All mice were cared for and handled according to the Guide for the Care and Use of Laboratory Animals published by the National Institutes of Health. Experimental protocol was approved by Shanghai Medical Experimental Animal Care Committee.

### AFP promoter assay

A SV40-hAFP promoter from pDrive-SV40-hAFP (InvivoGene) was chosen as the AFP promoter. The activity and tissue-specificity of the AFP promoter was assayed using GFP reporter in AFP-producing and non-AFP-producing cell lines. A recombinant lentivirus vector containing the AFP promoter and GFP reporter gene was constructed as follow. The AFP promoter was synthesized according to the instruction of the pDrive-SV40-hAFP with adding NheI and EcoRI restriction enzyme cutting sites (RECS) (See File S1). After amplification it was cloned into NheI-EcoRI sites of pLV-CMV-GFP lentiviral plasmid (MicroSCI, China) by replacing the CMV promoter. The recombinant lentiviral plasmid and the mother plasmid pLV-CMV-GFP were packaged by transient co-transfection of HEK 293 cells with helper-packaging plasmids (psPAX2 and pMD2.G, Trono Lab). The recombinant lentiviral vector was named as AFP-GFP while the mother vector was termed as CMV-GFP (served as positive control). To evaluate the activity of the AFP promoter, AFP-producing HCC cells were infected with either AFP-GFP (MOI = 5, 10, 20, 40 and 80) or CMV-GFP (MOI = 5). Three days later, the cells were observed under fluorescence microscope (Leica). The images were analyzed and the intensity of GFP fluorescence was quantitated by Image-Pro plus 6 software (MediaCybernetics). To evaluate the tissue-specificity of the AFP promoter, the HCCLM3, HepG2, Hep3B, L-02, HeLa, and SW1116 cells were all infected with AFP-GFP at MOI of 20. Three days later, the cells were observed and the GFP expression was quantified as mentioned above.

### Construction of AFP-miRNA and evaluation of RNAi efficacy

The AFP-miRNA targeting Beclin 1 was constructed as follow. Four miRNAs targeting Beclin 1 with negative control were designed and constructed into pcDNA6.2-GW/EmGFP-miR (Invitrogen). The vectors were named as pcDNA-miR-1, pcDNA-miR-2, pcDNA-miR-3, pcDNA-miR-4 and pcDNA-miR-NC. Then the 900 bp CMV-miRNA-EGFP structure was amplified from the templates pcDNA-miR-1/2/3/4/NC by PCR using primers Gecp-1,2 (Table 1). Then the CMV-miRNA-EGFP fragments were cloned into the NheI-NotI sites of a lentiviral vector pSil01 (MicroSCi, China) and formed new vectors (CMV-miRNA-1/2/3/4/NC). The HCCLM3 cells were infected with the CMV-miRNA-1/2/3/4/NC at MOI of 20. Q-PCR and western blot analysis of Beclin 1 gene silencing were performed to determine the most effective miRNA (CMV-miRNA-3). Then a 740 bp fragment A was amplified from template AFP-GFP by PCR using primers Gecp-3,4 (Table 1). A 230 bp fragment B was amplified from CMV-miRNA-3 or CMV-miRNA-NC by PCR using primers Gecp-5,6 (Table 1). A fragment C was generated from the templates fragment A and fragment B by PCR. Then the fragment C was cloned into the NheI-AvrII sites of the AFP-GFP and formed new vectors AFP-miRNA (AFP-miRNA-3/NC). The CMV-miRNA-3 was used as positive control. The AFP-miRNA-3/NC and CMV-miRNA-3/NC were then packaged into lentiviral particles. To evaluate the effectiveness of AFP-miRNA, the AFP-producing HCC cell lines (HCCLM3, HepG2, Hep3B) were infected with either CMV-miRNA-3 (MOI = 20) or AFP-miRNA-3 (MOI = 5, 10, 20, 40, 80, 160 and 320). Three days later, the cells were observed under fluorescence microscope (Leica). Q-PCR and western blot analysis of Beclin 1 gene silencing were performed one week later.

**Table 1:** Primers used for the construction of HCC-tissue specific RNAi systems.

Primer	Sequence
Gecp-1	CTAGAGCTAGCGCCACCATGGTGAGCAAGGGCGAGG
Gecp-2	ATCCTTGCGGCCGCTAGATATCTCGAGTGCGGCC
Gecp-3	TAACACGCTAGCGCCACCA
Gecp-4	GACGGCCACGAAGTGCTTAGCTTACTTGTACAGCTCGTCCATGC
Gecp-5	GCTAAGCACTTCGTGGCCGTC
Gecp-6	TCGACGCCTAGGGCGGCCGCTAGATATCTCGAGTGCGGCCA
Gecp-7	TTTTATCGATACTAGTGGCCTGAAATAACCTCTGAAAG
Gecp-8	CCTCTTCTTCTTGGGCATGGTGGCGTGTTATTGGCAGTGGTGG
Gecp-9	CATGCCCAAGAAGAAGAGGAAGGTGTCCAATTTACTGACCGTAC
Gecp-10	ATTCGCTAGCTCTAGACTAATCGCCATCTTCCAGCAG
Gecp-11	GGGCTCGAGCCCGGGAAGGTCGGGCAGGAAGAGGGCCTATTTCCCATGATT
Gecp-12	ATTACTTTCTACGTCACGTATTTTG
Gecp-13	TTTTAAAATGGACTATCATATGCTTACC
Gecp-14	AAGAATTCACGCGTGCATACCTGCGG
Gecp-15	CAAAATACGTGACGTAGAAAGTAATATAACTTCGTATAGCATACATTATAC
Gecp-16	AACTTCGTATAGCATACATTATACGAAGTTATGTTAACGTGGATAACCGTATTACCGCC
Gecp-17	CTTCGTATAATGTATGCTATACGAAGTTATGGATCCTTACTTGTACAGCTCGTCCATGC
Gecp-18	GGTAAGCATATGATAGTCCATTTTAAAAATAACTTCGTATAATGTATGCTATAC

The miRNA sequence: Beclin 1-F: TGCTGTAATGGAGCTGTGAGTTCCTGGTTTTGGCCACTGACTGACCAGGAACTCAGCTCCATTA; Beclin 1-R: CCTGTAATGGAGCTGAGTTCCTGGTCAGTCAGTGGCCAAAACCAGGAACTCACAGCTCCATTAC.

### Construction of AFP-Cre/LoxP-shRNA system and evaluation of effectiveness and tissue-specificity

The AFP-Cre/LoxP-shRNA system consists of AFP-Cre and LoxP-shRNA lentiviral vectors. The AFP-Cre vector contains a Cre gene driven by the AFP promoter. The LoxP-shRNA vector has a modified U6 promoter followed by shRNA against target gene (Beclin 1). The modified U6 promoter harbors a LoxP-CMV-eGFP-LoxP inside. When the AFP-Cre and LoxP-shRNA vectors co-infect target cells, the AFP promoter will drive the expression of Cre recombinase which subsequently cuts the LoxP-CMV-eGFP-LoxP inside the U6 promoter and activates the U6 promoter. The activated U6 promoter then drives the down-stream shRNA expression and silences the target gene. The CMV-eGFP inside the U6 promoter serves as an indicator (when the CMV-eGFP is cut by the Cre recombinase, the GFP fluorescence will diminish or disappear). The AFP-Cre and LoxP-shRNA vectors were constructed as follow: *(1) AFP-Cre vector*: The pCDH-CMV-MCS-EF1-Puro (SBI) was used to generate the AFP-Cre. The AFP promoter fragment was amplified from the template AFP-GFP by PCR using primer Gecp-7,8 (Table 1). The Cre (NLS-Cre) was amplified from the template pLV-CRE (MedSCI, China) using primer Gecp-9,10 (Table 1). The AFP-Cre structure fragment was generated from the template AFP promoter and Cre by PCR using primer Gecp-7,10 (Table 1). The AFP-Cre structure (See File S2) was then cloned into the SpeI-XbaI sites of pCDH-CMV-MCS-EF1-Puro by In-Fusion cloning technique (Clontech) and formed the AFP-Cre vector. *(2) LoxP-shRNA vector*: Fragment A and fragment B were cloned from template pSil02 vector (MicroSCI, China) by PCR using primers Gecp-11,12 and Gecp-13,14 (Table 1), respectively. A fragment C was generated by PCR from template pSil04 (MicroSCI, China) using primers Gecp-15,16,17,18 (Table 1). A fragment D (U-LoxP-CMV-eGFP-U6 structure, See File S2) was generated by PCR from templates fragments A, B, C using primers Gecp-11,14 (Table 1). The fragment D was then cloned into the XhoI-EcoRI sites of the pSil02 vector and formed the LoxP-shRNA vector. A previously validated shRNA targeting Beclin 1 (See File S3) was cloned into the AgeI-EcoRI sites of LoxP-shRNA vector. The AFP-Cre and LoxP-shRNA were then separately packaged into lentiviral particles. The effectiveness and tissue-specificity of the AFP-Cre/LoxP-shRNA system were examined *in vitro* and *in vivo*. *(1)In vitro evaluation*: The AFP-producing HCC cells (HCCLM3/HepG2/Hep3B) and non-AFP-producing cells (L-02/Hela/SW1116) were infected with the AFP-Cre/LoxP-shRNA system targeting Beclin 1 (AFP-Cre/LoxP-shRNA-Beclin1) (AFP-Cre:LoxP-shRNA = 1, MOI = 1,5,10,20 for each). The cells were observed under fluorescence microscope every day. Q-PCR and western blot analysis of Beclin 1 gene silencing were performed one week later. *(2)In vivo evaluation*: Xenograft nude mouse model of HCC via orthotopic implantation and subcutaneous inoculation of HCCLM3 cells were established as previously described [19]. *Intravenous injection*: Twelve mice were randomly divided into two groups (n = 6 per group). One week after orthotopic implantation, the AFP-Cre/LoxP-shRNA system was intravenously injected via tail vein (*LoxP-shRNA group*: LoxP-shRNA 1.8×10^8^ TU in 180 µl Opti-MEM; *Cre+LoxP group*: AFP-Cre 0.9×10^8^ TU+LoxP-shRNA 0.9×10^8^ TU in 180 µl Opti-MEM). The mice were sacrificed two weeks later. *Intratumoral injection*: Thirty-six mice were randomly divided into four groups (n = 6 per group). When the subcutaneous tumors reached a size of about 4 mm maximal diameter, the AFP-Cre/LoxP-shRNA system was intratumorally injected (*OMEM group*: 50 µl Opti-MEM; *AFP-Cre group*: 1×10^8^ TU AFP-Cre in 50 µl Opti-MEM; *LoxP-shRNA group*: 1×10^8^ TU LoxP-shRNA in 50 µl Opti-MEM; *Cre+LoxP group 1*: 0.25×10^8^ TU AFP-Cre+0.25×10^8^ TU LoxP-shRNA vectors in 50 µl Opti-MEM; *Cre+LoxP group 2*: 0.5×10^8^ TU AFP-Cre+0.5×10^8^ TU LoxP-shRNA vectors in 50 µl Opti-MEM). All mice were sacrificed two weeks later. All of the tumors were resected. The frozen sections of the tumors were stained with DAPI (Invitrogen) and observed under fluorescence microscope as mentioned below. Q-PCR and Western blot analysis of Beclin 1 silencing were performed.

The Beclin 1 shRNA sequence: Beclin 1-F: CCGGCCCGTGGAATGGAATGAGATTCTCGAGAATCTCATTCCATTCCACGGGTTTTTG;Beclin 1-R: AATTCAAAAACCCGTGGAATGGAATGAGATTCTCGAGAATCTCATTCCATTCCACGGG.

### Quantitative real-time PCR analysis

The quantitative real-time PCR (Q-PCR) analysis of Atg5 and Beclin 1 expression was performed as previously described [22].

### Western blot analysis

Western blot analysis was performed as previously described [22]. The following antibodies were used: anti-human antibodies against Atg5 (1∶500; Cell Signaling), Beclin 1 (1∶1000; Cell Signaling), or glyceraldehyde-3-phosphate dehydrogenase (GAPDH, 1∶5000; Millipore).

### Cell viability assay

Cell viability was determined with WST-8 cytotoxicity assay using Cell Counting Kit-8 (Dojindo, Japan) as previously described [23].

### Fluorescence microscopy of tissues

After the mice were killed, the tumors were resected immediately and embedded in Tissue-Tek OCT compound using liquid nitrogen and stored at −80°C. Then the tissue samples were sectioned at 40 µm thickness with a cryostat. The tissue sections were stained with DAPI (1∶1000 dilution, 15 min; Invitrogen). Then they were observed and analyzed using confocal fluorescence microscope (Carl Zeiss).

### Construction of AFP-Cre/LoxP-shRNA targeting Atg5 and evaluation of its efficacy for sensitizing HCC cells to sorafenib treatment in vitro and in vivo

A previously validated Atg5 shRNA (See File S3) was cloned into the AFP-Cre/LoxP-shRNA system in a similar fashion as mentioned above and formed the AFP-Cre/LoxP-shRNA targeting Atg5 gene (AFP-Cre/LoxP-shRNA-Atg5). The AFP-producing HCC cells (MHCC97L and HepG2) were infected with AFP-Cre/LoxP-shRNA-Atg5 (MOI = 1, 5, 10 and 20). Q-PCR and western blot analysis of Atg5 gene silencing were performed one week later. The AFP-Cre/LoxP-shRNA-Atg5 -mediated sensitization of HCC cells to sorafenib treatment was evaluated *in vitro* and *in vivo*. *(1)In vitro evaluation:* The MHCC97-L and PLC/PRF/5 cells were infected with the AFP-Cre/LoxP-shRNA-Atg5 (AFP-Cre:LoxP-shRNA = 1, MOI = 20 for each). One week later, the virus-infected cells were exposed to sorafenib (20 µM, Bayer) for 24 h. Cells without infection and cells infected with AFP-Cre, LoxP-shRNA, or AFP-Cre/LoxP-shRNA-NC served as controls. Apoptosis was measured using Annexin V and PI flow cytometry as previously described [23]. *(2)In vivo evaluation:* Xenograft nude mouse model of HCC via subcutaneous inoculation of MHCC97-L cells (1×10^7^) was established as previously described [24]. Twelve mice were randomly divided into two groups (n = 6 per group): (i) Sorafenib group (sorafenib treatment alone); (ii) Sorafenib+Cre/LoxP group (AFP-Cre/LoxP-shRNA-Atg5 treatment followed by sorafenib treatment). The AFP-Cre/LoxP-shRNA-Atg5 treatment alone was not included as pilot studies showed that the AFP-Cre/LoxP-shRNA-Atg5 treatment had no effect on the tumorigenesis of MHCC97L cells (see File S4). Tumor size was determined by caliper measurements every 3 days. When the subcutaneous tumors reached a size of about 4 mm maximal diameter, the mice in the Sorafenib+Cre/LoxP group were treated with the AFP-Cre/LoxP-shRNA-Atg5 by intratumorally injection (0.5×10^8^ TU AFP-Cre+0.5×10^8^ TU LoxP-shRNA-Atg5 in 50 µl Opti-MEM). One week after AFP-Cre/LoxP-shRNA-Atg5 treatment, all mice in the Sorafenib group and Sorafenib+Cre/LoxP group were treated daily with sorafenib (30 mg/kg) via intraperitoneal injection. The animals were monitored every day and sacrificed 6 weeks after tumor implantation. All of the tumors were resected and the tumor weights were measured.

The Atg5 shRNA sequence: Atg5-F: CCGGGCTAGCTGGCTGTCCATATTTCAAGAGAATATGGACAGCCAGCTAGCTTTTTTG;Atg5-R: AATTCAAAAAAGCTAGCTGGCTGTCCATATTCTCTTGAAATATGGACAGCCAGCTAGC.

### Statistical Analysis

Statistical analysis was performed with SPSS 13.0 software (SPSS, Chicago, IL). Results were presented as mean ± standard deviation (SD). Comparisons of quantitative data were analyzed using Student's *t* test between two groups or by one-way ANOVA for multiple groups. *P* values<0.05 were considered statistically significant.

## Results

### AFP-promoter is active and specific in AFP-producing HCC cells and tissues

A recombinant lentiviral vector containing GFP reporter gene driven by AFP promoter was constructed (AFP-GFP) (Fig. 1A). The activity and tissue-specificity of the AFP promoter were assayed by infecting the AFP-producing and non-AFP-producing cells with the AFP-GFP vector. GFP reporter assay showed that the AFP-promoter could efficiently drive GFP expression in AFP-producing HCC cells (HepG2, Hep3B, and HCCLM3) but not in non-HCC cells (L-02, SW1116, and Hela) (Fig. 1B,D). The GFP expression was vector dose-dependent (Fig. 1 C,E). However, as compared with the CMV promoter which is known to be one of the strongest promoters in a wide range of cell lines, the transcriptional activity of the AFP promoter was remarkably lower (Fig. 1E).

**Figure 1:** Activity and tissue-specificity of the AFP promoter. (A) Construction of recombinant lentiviral vectors containing GFP reporter gene driven by AFP promoter or CMV promoter (AFP-GFP and CMV-GFP) for AFP promoter assay. (B,D) The AFP promoter is active and HCC tissue-specific. GFP was highly expressed in AFP-producing HCC cells (HepG2, Hep3B, and HCCLM3) but not in non-HCC cells (normal hepacyte L-02, cervical cancer cell Hela, and colon cancer cell SW1116). (C,E) The AFP promoter was efficient for transgenic expression but its activity was weaker than CMV-promoter, as exemplified by HCCLM3 cells infected with AFP-GFP (MOI = 5–80) and CMV-GFP (MOI = 5).

### AFP-miRNA system can silence target gene but requires high titer

We first investigated the strategy of AFP-promoter driven miRNA for HCC-specific gene silencing. An AFP-miRNA lentiviral vector (AFP-miRNA) targeting Beclin 1 gene was constructed (Fig. 2A). A CMV promoter driven miRNA vector (CMV-miRNA) served as positive control (Fig. 2A). To assess the effectiveness of the AFP-miRNA, AFP-producing HCC cells (HCCLM3, HepG2, and Hep3B) were infected with the AFP-miRNA at various MOI. The AFP-miRNA was efficient in infecting all cell lines *in vitro* (Fig. 2B). Q-PCR and western blot analysis of Beclin 1 gene silencing showed that the AFP-miRNA could knockdown Beclin 1 but required considerably high titer (Fig. 2C). A MOI of more than 80 was required to achieve efficient gene silencing (Fig. 2C). As compared with positive control CMV-miRNA, the efficacy of the AFP-miRNA was remarkably weaker (Fig. 2C). The CMV-miRNA infection at a MOI of 20 could achieve silencing level equal to that of the AFP-miRNA infection at a MOI of 320 in AFP-producing HCC cells (Fig. 2C). As high titer was needed for effective gene silencing, the cytotoxicity of the AFP-miRNA against target cells was determined. Cell viability assay showed that the AFP-miRNA infection at required titer (MOI>80) led to considerable cell death. With the increase of MOI, the cytotoxicity significantly enhanced (Fig. 2D).

**Figure 2:** Effectiveness of AFP-miRNA system for HCC tissue-specific RNAi. (A) Construction of recombinant lentiviral vectors contained miRNA targeting Beclin 1 gene driven by AFP promoter or CMV promoter (AFP-miRNA and CMV-miRNA). (B) The AFP-miRNA system could efficiently infected HCC cells (more than 99%), as exemplified by HCCLM3 cells. (C) Q-PCR and western blot analysis showed that the AFP-miRNA system could downregulate target gene (Beclin 1) of HCC cells but required high titer (MOI>80), as compared with positive control CMV-miRNA. (D) Cell viability assay showed that the high titer required for effective AFP-miRNA-mediated RNAi was cytotoxic to target HCC cells, as exemplified by HCCLM3 and HepG2 cells.

As the AFP-miRNA required a high titer which was cytotoxic to target cells, it was not desirable for target therapy because it might cause damage to the adjacent normal cells and tissues. Therefore, another system (AFP-Cre/LoxP-shRNA) was constructed (Fig. 3A).

**Figure 3:** Effectiveness and tissue-specificity of AFP-Cre/LoxP-shRNA system for HCC tissue-specific RNAi. (A) Construction of the AFP-Cre/LoxP-shRNA system which consists of AFP-Cre and LoxP-shRNA vectors. (B) Schematic illustration of the AFP-Cre/LoxP-shRNA system. When the AFP-Cre and LoxP-shRNA vectors co-infect target cells, the AFP promoter drives the downstream Cre recombinase gene expression which subsequently cuts the LoxP-CMV-eGFP-LoxP inside the U6 promoter and activates it. The activated U6 promoter then drives the downstream shRNA expression. The LoxP-shRNA harbors a CMV-eGFP indicator which can indicate the RNAi expression (GFP fluorescence will diminish if the AFP promter initiates the RNAi expression). (C, D) CMV-eGFP indicator and gene silencing analysis by Q-PCR and western blot showed that the AFP-Cre/LoxP-shRNA system targeting Beclin 1 (AFP-Cre/LoxP-shRNA-Beclin1) could efficiently silence target gene (Beclin 1) in a HCC-specific manner. The GFP fluorescence diminished in HCC cells (HCCLM3, HepG2, and Hep3B) but not in non-HCC cells (L-02, Hela, and SW1116) after infection with the AFP-Cre/LoxP-shRNA-Beclin1. Q-PCR and western blot analysis were exemplified by HCC cell line HCCLM3 and non-HCC cell line L-02.

### AFP-Cre/LoxP-shRNA system can efficiently silence target gene in a HCC-specific manner

The AFP-Cre/LoxP-shRNA system was successfully established (Fig. 3A). The CMV-eGFP indicator inside could well indicate whether the system worked as desired (Fig. 3B,C). The GFP fluorescence diminished after AFP-Cre and LoxP-shRNA co-infected AFP-producing HCC cells (HCCLM3, HepG2, and Hep3B) while it did not change as AFP-Cre and LoxP-shRNA infected the non-HCC cells (L-02, Hela, and SW1116) (Fig. 3C). To assess the effectiveness and tissue-specificity of the AFP-Cre/LoxP-shRNA system, AFP-producing HCC cells (HCCLM3, HepG2, and Hep3B), normal hepatocyte (L-02), and non-HCC cancer cells (Hela and SW1116) were infected with the AFP-Cre/LoxP-shRNA system at a MOI of 1,5,10 or 20. Q-PCR and western blot analysis showed that the system could efficiently silence Beclin 1 gene in only AFP-producing HCC cells (Fig. 3C,D). It could effectively knockdown target gene at a MOI of 10–20 instead of the high titer required for the AFP-miRNA system (Fig. 3D). The effectiveness of the system was further examined *in vivo*. Systemic administration of the AFP-Cre/LoxP-shRNA system was firstlytested. Nude mouse model of HCC via orthotopic implantation was established using AFP-producing HCC cells (HCCLM3) and the AFP-Cre/LoxP-shRNA-Beclin1 was intravenously injected (Fig. 4B). Q-PCR and western blot analysis indicated that there was no significant decrease of Beclin 1 gene after the AFP-Cre/LoxP-shRNA-Beclin1 was given (Fig. 4A). Intravenous injection of LoxP-shRNA with CMV-eGFP indicator showed no GFP expression in HCC tumor, which suggested that no vectors were delivered into the tumor cells (Fig. 4B). The ineffectiveness of systemic administration was thought to be attributed to the disadvantages of the nude mouse model and lentivirus-based vector. The effectiveness of in vivo application of the system was then examined by intratumorally administration. Nude mouse model of HCC via subcutaneous injection was established using HCCLM3 cells (Fig. 4D). The AFP-Cre/LoxP-shRNA-Beclin1 was intratumorally injected into the subcutaneous tumor. The GFP indicator analysis showed that the system could efficiently infect HCC cells (Fig. 4D). Q-PCR and western blot analysis showed that it could efficiently knockdown the Beclin 1 gene of the HCCLM3 tumor tissues *in vivo* (Fig. 4C).

**Figure 4:** Efficacy of AFP-Cre/LoxP-shRNA system for HCC tissue-specific RNAi *in vivo*. (A,B) Mouse model of HCC via orthotopic implantation of HCCLM3 cells was established. Q-PCR and western blot analysis showed that intravenous injection of the AFP-Cre/LoxP-shRNA-Beclin1 did not knockdown Beclin 1 gene. GFP indicator analysis showed no GFP expression after the LoxP-shRNA vector was intravenously given, suggesting that the system did not enter the tumor in the liver. (C,D) Mouse model of HCC via subcutaneous inoculation of HCCLM3 cells was established. Q-PCR and western blot analysis showed that intratumoral injection of the AFP-Cre/LoxP-shRNA-Beclin1 could efficiently silence target gene (Beclin 1) *in vivo*. GFP indicator indicated that the AFP-Cre/LoxP-shRNA could efficiently infect and work in HCC tissue *in vivo* (GFP fluorescence diminished after intratumoral injection of the AFP-Cre/LoxP-shRNA, the LoxP-shRNA alone served as control). (Cre+LoxP: infection of AFP-Cre/LoxP-shRNA-Beclin1; AFP-Cre and LoxP-shRNA: infection of AFP-Cre or LoxP-shRNA alone).

### AFP-Cre/LoxP-shRNA-Atg5 mediated Atg5 silencing sensitizes HCC cells or tissues to sorafenib-mediated lethality

Our previous study showed that silencing of Atg5 gene could enhance sorafenib-mediated lethality [18]. We next used the Atg5 as target gene to validate the effectiveness of the AFP-Cre/LoxP-shRNA system and test the value of the system for HCC treatment. The AFP-Cre/LoxP-shRNA system targeting Atg5 (AFP-Cre/LoxP-shRNA-Atg5) was successfully constructed. Q-PCR and western blot analysis showed that the AFP-Cre/LoxP-shRNA-Atg5 could efficiently downregulate Atg5 in AFP-producing cells (MHCC97L and PLC) (Fig. 5A). We then examined whether the AFP-Cre/LoxP-shRNA-Atg5 could sensitize HCC cells to sorafenib treatment. The efficacy of the AFP-Cre/LoxP-shRNA-Atg5 was firstly examined *in vitro*. Apoptosis assay showed that the apoptotic rate of cells (MHCC97L and PLC) treated with AFP-Cre/LoxP-shRNA-Atg5 plus sorafenibwas significantly higher than that of cells receiving sorefenib alone (all *P*<0.05) (Fig. 5B). To further evaluate whether the AFP-Cre/LoxP-shRNA system can be translated into a practical therapeutic modality, the AFP-Cre/LoxP-shRNA-Atg5 was next tested *in vivo*. A nude mouse model of HCC was established using MHCC97L cells and the AFP-Cre/LoxP-shRNA-Atg5 was intratumorally administrated. Q-PCR and western blot analysis showed that the AFP-Cre/LoxP-shRNA-Atg5 could efficiently downregulate Atg5 *in vivo* (Fig. 5C). The average tumor weight of mice receiving AFP-Cre/LoxP-shRNA-Atg5 plus sorafenib (1.04±0.33) was significantly lower than that of mice subjected to sorafenib alone (1.42±0.29) (*P* = 0.039) (Fig. 5D). These results indicated that the AFP-Cre/LoxP-shRNA-Atg5 could enhance sorafenib treatment.

**Figure 5:** Application of AFP-Cre/LoxP-shRNA targeting Atg5 gene for enhancement of sorafenib treatment. (A) Construction of the AFP-Cre/LoxP-shRNA system targeting Atg5 gene (AFP-Cre/LoxP-shRNA-Atg5). Q-PCR and western blot analysis showed that it could efficiently knockdown Atg5 gene. (B) Combination of AFP-Cre/LoxP-shRNA-Atg5 infection and sorafenib treatment induced a significantly increase in apoptosis of HCC cells (MHCC97L and PLC) as compared to sorafenib treatment alone. Apoptosis was quantified by annexin V/PI FCM analysis. (C) Q-PCR and western blot analysis showed that intratumoral injection of the AFP-Cre/LoxP-shRNA-Atg5 efficiently silenced Atg5 gene *in vivo*. (D) The AFP-Cre/LoxP-shRNA-Atg5 significantly enhanced sorafenib-induced suppression of tumorigenicity of MHCC97L cells *in vivo*. The tumor weight of mice receiving intratumoral injection of the AFP-Cre/LoxP-shRNA-Atg5 combined with sorafenib was significantly lower than that of mice subjected to sorafenib alone. (Cre+LoxP: infection of AFP-Cre/LoxP-shRNA-Atg5; AFP-Cre and LoxP-shRNA: infection of AFP-Cre or LoxP-shRNA alone). (*P<0.05, **P<0.01).

## Discussion

In this study, an efficient HCC tissue-specific RNAi system (AFP-Cre/LoxP-shRNA) was successfully established. *In vitro* and *in vivo* analysis showed that it could efficiently silence target gene in an HCC-specific manner. Application of the system targeting Atg5 was shown to be able to enhance sorafenib treatment *in vitro* and *in vivo*, suggesting its value for HCC therapy. Our system provides a usable tool for HCC tissue-specific RNAi therapy, which holds significant promise as new approach for the management of HCC.

In recent years, with tremendous advance in HCC research, increasing HCC-related genes have been discovered. Translating these findings into clinical therapy, especially target therapy, holds great promise for HCC treatment [1], [6], [7]. The RNAi is a powerful tool for gene silencing. It can exert target therapy while avoid off-target side-effects. Increasing evidence shows that RNAi has great potential to be developed into HCC therapy [7], [17]. However, some obstacles must be overcome before the successful therapeutic application. [4]. RNAi should be capable of sustained inhibition of target gene while exerting its effect within target cells or tissues. With regard to targeting cells or tissues of interest, there are two strategies, including envelope-mediated entry targeting strategy and tissue-specific promoter -mediated targeting strategy [17]. (1) Envelope-mediated entry targeting strategy. Combining viral particles with a foreign envelope glycoprotein can alter the host tropism of viral vector. Using the hepatic virus envelope glycoprotein to pseudotype the host tropism and generate HCC tissue-type viral vectors may obtain targeting RNAi to HCC tissues; (2) Tissue-specific promoter -mediated targeting strategy. Using a tissue-specific promoter as an internal promoter can target expression to the cells of interest. Unlike the pseudotyping vectors in envelope-mediated strategy, vectors with a tissue-specific promoter can basically enter and integrate in any cell types. But their expression is limited to a certain cell type by the internal promoter. Various tissue-specific promoters have been incorporated into lentiviral vectors, including the AFP promoter [17]. Given the more complex structure of the envelop-mediated target delivery and difficulty de novo design, we chose to use HCC specific promoter (AFP-promoter) in combination with lenti vector to construct the RNAi system required. The AFP promoter is a commonly used HCC tissue-specific promoter because of its high specificity. It has been used to drive therapeutic genes expression to achieve HCC-specific target therapy [11]–[16]. Lenti vector-mediated RNAi is a powerful method for persistent and specific gene silencing. RNAi can be triggered by microRNA (miRNA) or small interfering RNA (siRNA) [7]. Regarding lentiviral vectors, RNAi can be delivered as shRNA driven by a Pol III promoter (such as U6) or microRNA (miRNA) expressed from a Pol II promoter (such as CMV or tissue-specific promoter) [7], [17]. The lentivirus-delivered shRNA or miRNA can be stably integrated into the target cell genome, allowing permanent and heritable gene silencing [17]. In this study, we designed two systems, including miRNA-based AFP-miRNA and shRNA-based AFP-Cre/LoxP-shRNA. The miRNA can be directly driven by Pol II promoter. We firstly tested whether the AFP promoter (Pol II) could drive miRNA expression to obtain effective RNAi. Our data showed that the AFP-miRNA could decrease target gene but required a high titer that was lethal to target cells, which excluded the *in vivo* application as it posed threat to adjacent normal cells or tissues. The low efficacy of the AFP-miRNA was attributed to the weak activity of the AFP promoter. Although the AFP promoter was shown to able to drive GFP expression, the transcriptional activity appeared to be insufficient to mediate efficient miRNA expression. As the AFP-miRNA could not achieve satisfatory efficacy, we then attempted the shRNA strategy. The shRNA cannot be directly driven by the AFP promoter (Pol II) but it can be efficiently driven by Pol III promoter (such as U6). However, the Pol III promoters mediated RNAi cannot be controlled in a tissue-specific manner because the Pol III promoters are constitutively expressed in all cell types. To circumvent this problem, a switch structure (Cre/loxP system combined with a modified U6 promoter) was designed to obtain shRNA expression driven by AFP promoter. Our results strongly demonstrated that the novel system could efficiently mediate shRNA expression and specifically silence target gene of HCC cells or tissues. Further application of the system for HCC treatment showed that the system was valuable for HCC therapy. The system-mediated HCC-specific Atg5 silencing enhanced sorafenib treatment. Although the Atg5 gene was shown to be not an optimal target gene for HCC RNAi therapy as its efficacy was weak, the validation using Atg5 had demonstrated the value of the AFP-Cre/LoxP-shRNA system. With the application of new better target gene, a satisfactory effect of the system-mediated RNAi therapy will be achieved.

Although the AFP-Cre-LoxP-shRNA system is shown efficient for HCC tissue-specific RNAi, it still carries some inherent disadvantages. The main one is that intravenous application of the system appears to be ineffective. This is not consistent with our expectations. The systemic administration of the system was thought to be able to achieve satisfactory efficacy since numerous studies had demonstrated that RNAi agents (siRNAs) could be easily delivered into the liver and liver tumor was suitable for intravenous application [7]. However, our data showed that intravenous injection of the system was not effective. This may be due to several reasons. First, intake of the system is limited. Due to the limitations of the lentiviral vector (maximum concentration is 2×10^9^ TU/ml) and the nude mouse model (maximum volume of intravenous injection is 180 µl), the maximum intake is only 3.6×10^8^ TU. Second, there is a considerable loss of the system during intravenous administration. The lentivrial vector used for this study has a wide host tropsin. It can quickly transfect any type of cells, although it works in only AFP-producing HCC cells. After being intravenously injected, it may immediately infect blood, endothelial cells or any other cells it encountered and then is considerably consumed before it reaches the tumor in the liver. The commonly used hydrodynamic injection was not used in this study. Although it is an effective way of delivering therapeutic agents into the liver in HCC mouse models [25], [26], this delivery method is found to be associated with significant mortality in our pilot study, which excluded it from systemic application as human HCC therapy was the final objective. Significant efforts are still required to improve the current system. The vector manipulation may be a possible solution. Lentiviral vector is a system easy to be manipulated [17]. Limiting the lentiviral vector entry through pseudotyping with heterologous viral glycoproteins is a practical strategy. Using the hepatic virus envelope glycoprotein for pseudotyping the host tropism to generate HCC tissue-type lentivectors may obtained targeted delivery of RNAi to HCC tissues and efficiently overcome the biological barriers. The vector manipulation is under investigation and the promising result is expected to be presented in the future.

Taken together, in this study, an HCC tissue-specific RNAi system (AFP-Cre/LoxP-shRNA) was successfully developed. The AFP-Cre/LoxP-shRNA system can efficiently silence target gene in an HCC tissue-specific manner. The system mediated silencing of therapeutic gene is valuable as adjuvant therapy for HCC treatment. Our system provides a usable tool for HCC-specific RNAi therapy, which may serve as a new therapeutic modality for the management of HCC.

## Supporting Information

File S1 The sequence of AFP promoter.
(DOC)

File S2 The AFP-Cre structure and U-LoxP-CMV-eGFP-LoxP-U6 structure.
(DOC)

File S3 Determination of the effective shRNAs targeting Beclin 1 and Atg5.
(DOC)

File S4 Comparison of the effects of AFP-Cre/LoxP-shRNA-Atg5 among sorafenib alone, and Cre/PoxP with and without sorafenib treatment.
(DOC)

## References

[1] FornerA, LlovetJM, BruixJ (2012) Hepatocellular carcinoma. Lancet 379: 1245–1255.2235326210.1016/S0140-6736(11)61347-0PMC13537732

[2] DavisME, ZuckermanJE, ChoiCHJ, SeligsonD, TolcherA, et al (2010) Evidence of RNAi in humans from systemically administered siRNA via targeted nanoparticles. Nature 464: 1067–1070.2030563610.1038/nature08956PMC2855406

[3] PecotCV, CalinGA, ColemanRL, Lopez-BeresteinG, SoodAK (2011) RNA interference in the clinic: challenges and future directions. Nat Rev Cancer 11: 59–67.2116052610.1038/nrc2966PMC3199132

[4] ChenSH, ZhaoriG (2011) Potential clinical applications of siRNA technique: benefits and limitations. Eur J Clin Invest 41: 221–232.2096468010.1111/j.1365-2362.2010.02400.x

[5] PetroccaF, LiebermanJ (2011) Promise and challenge of RNA interference-based therapy for cancer. J Clin Oncol 29: 747–754.2107913510.1200/JCO.2009.27.6287

[6] MarquardtJU, GallePR, TeufelA (2012) Molecular diagnosis and therapy of hepatocellular carcinoma (HCC): an emerging field for advanced technologies. J Hepatol 56: 267–275.2178275810.1016/j.jhep.2011.07.007

[7] XuC, LeeSA, ChenX (2011) RNA interference as therapeutics for hepatocellular carcinoma. Recent Pat Anticancer Drug Discov 6: 106–115.2111082710.2174/157489211793980097

[8] BoraRS, GuptaD, MukkurTK, SainiKS (2012) RNA interference therapeutics for cancer: Challenges and opportunities (Review). Mol Med Report 6: 9–15.10.3892/mmr.2012.87122576734

[9] GilmoreIR, FoxSP, HollinsAJ, AkhtarS (2006) Delivery strategies for siRNA-mediated gene silencing. Curr Drug Deliv 3: 147–145.1661100110.2174/156720106776359159

[10] JohnsonPJ (1999) Role of alpha-fetoprotein in the diagnosis and management of hepatocellular carcinoma. J Gastroenterol Hepatol 14 Suppl: S32–36.1038263610.1046/j.1440-1746.1999.01873.x

[11] IdoA, NakataK, KatoY, NakaoK, MurataK, et al (1995) Gene therapy for hepatoma cells using a retrovirus vector carrying herpes simplex virus thymidine kinase gene under the control of human alpha-fetoprotein gene promoter. Cancer Res 55: 3105–3109.7541712

[12] KanekoS, TamaokiT (2001) Gene therapy vectors harboring AFP regulatory sequences. Preparation of an adenoviral vector. Mol Biotechnol 19: 323–330.1172162810.1385/MB:19:3:323

[13] HiranoT, KanekoS, KanedaY, SaitoI, TamaokiT, et al (2001) HVJ-liposome-mediated transfection of HSVtk gene driven by AFP promoter inhibits hepatic tumor growth of hepatocellular carcinoma in SCID mice. Gene Ther 8: 80–83.1140230610.1038/sj.gt.3301355

[14] KanaiF, LanKH, ShiratoriY, TanakaT, OhashiM, et al (1997) In vivo gene therapy for alpha-fetoprotein-producing hepatocellular carcinoma by adenovirus-mediated transfer of cytosine deaminase gene. Cancer Res 57: 461–465.9012474

[15] MaoCY, HuaHJ, ChenP, YuDC, CaoJ, et al (2009) Combined use of chemotherapeutics and oncolytic adenovirus in treatment of AFP-expressing hepatocellular carcinoma. Hepatobiliary Pancreat Dis Int 8: 282–287.19502169

[16] TakahashiM, SatoT, SagawaT, LuY, SatoY, et al (2002) E1B-55K-deleted adenovirus expressing E1A-13S by AFP-enhancer/promoter is capable of highly specific replication in AFP-producing hepatocellular carcinoma and eradication of established tumor. Mol Ther 5: 627–634.1199175410.1006/mthe.2002.0589

[17] SakumaT, BarryMA, IkedaY (2012) Lentiviral vectors: basic to translational. Biochem J 443: 603–618.2250712810.1042/BJ20120146

[18] ShiYH, DingZB, ZhouJ, HuiB, ShiGM, et al (2011) Targeting autophagy enhances sorafenib lethality for hepatocellular carcinoma via ER stress-related apoptosis. Autophagy 7: 1159–1172.2169114710.4161/auto.7.10.16818

[19] LiY, TangY, YeL, LiuB, LiuK, et al (2003) Establishment of a hepatocellular carcinoma cell line with unique metastatic characteristics through in vivo selection and screening for metastasis-related genes through cDNA microarray. J Cancer Res Clin Oncol 129: 43–51.1261890010.1007/s00432-002-0396-4PMC12161897

[20] LiY, TangZ-Y, HouJ-X (2012) Hepatocellular carcinoma: insight from animal models. Nat Rev Gastroenterol Hepatol 9: 32–43.10.1038/nrgastro.2011.19622025031

[21] LiY, TangZY, YeSL, LiuYK, ChenJ, et al (2001) Establishment of cell clones with different metastatic potential from the metastatic hepatocellular carcinoma cell line MHCC97. World J Gastroenterol 7: 630–636.1181984410.3748/wjg.v7.i5.630PMC4695564

[22] DingZB, ShiYH, ZhouJ, QiuSJ, XuY, et al (2008) Association of autophagy defect with a malignant phenotype and poor prognosis of hepatocellular carcinoma. Cancer Res 68: 9167–9175.1901088810.1158/0008-5472.CAN-08-1573

[23] PengY, ZhengM, FengB, ChenX, YuB, et al (2008) Hyperthermic CO2 pneumoperitoneum induces apoptosis in human colon cancer cells through Bax-associated mitochondrial pathway. Oncol Rep 19: 73–79.18097578

[24] LiY, TianB, YangJ, ZhaoL, WuX, et al (2004) Stepwise metastatic human hepatocellular carcinoma cell model system with multiple metastatic potentials established through consecutive in vivo selection and studies on metastatic characteristics. J Cancer Res Clin Oncol 130: 460–468.1514632910.1007/s00432-004-0564-9PMC12161865

[25] YangPL, AlthageA, ChungJ, ChisariFV (2002) Hydrodynamic injection of viral DNA: a mouse model of acute hepatitis B virus infection. Proc Natl Acad Sci U S A 99: 13825–13830.1237486410.1073/pnas.202398599PMC129782

[26] ZhangG, GaoX, SongYK, VollmerR, StolzDB, et al (2004) Hydroporation as the mechanism of hydrodynamic delivery. Gene Ther 11: 675–682.1472467310.1038/sj.gt.3302210PMC4412368

